# Significance of B10 cell in patients with thymoma complicated with myasthenia gravis

**DOI:** 10.18632/oncotarget.17908

**Published:** 2017-05-17

**Authors:** Yang Lu, Fanjie Meng, Yang Yang, Lan Li, Donghao Wang, Yuantao Cui, Shangwen Dong, Wanhua Wang

**Affiliations:** ^1^ Department of Intensive Care Unit, Tianjin Medical University Cancer Institute and Hospital, National Clinical Research Center for Cancer, Key Laboratory of Cancer Prevention and Therapy, Tianjin, Tianjin's Clinical Research Center for Cancer, Tianjin, 300060, China; ^2^ Department of Cardiothoracic Surgery, Tianjin Medical University General Hospital, Tianjin, 300052, China; ^3^ Department of Anesthesia, Tianjin Medical University Cancer Institute and Hospital, National Clinical Research Center for Cancer, Key Laboratory of Cancer Prevention and Therapy, Tianjin, Tianjin's Clinical Research Center for Cancer, Tianjin, 300060, China; ^4^ Key Laboratory of Pharmacology of Traditional Chinese Medicine Formulae, Ministry of Education, Tianjin University of Traditional Chinese Medicine, Tianjin, 300193, China

**Keywords:** regulatory B cell, B10 cell, thymoma, myasthenia gravis, autoimmune abnormality

## Abstract

A subset of regulatory B cells in humans has been identified as B10 cell which has the function of secreting interleukin-10. We evaluated the significance of B10 cell in patients with thymoma complicated with myasthenia gravis. In this study, 156 patients diagnosed with thymoma were enrolled, FCM was used to detected the percentage of Breg/CD19^+^B cells and CD19^+^B cells/PBMC, ELISA to evaluate the serum concentration of the relevant immunological markers; purified CD19^+^B cells in tissues by MACS; gene and protein expressions of CD19 and IL-10 by Real-time PCR and Western-Blot; double immunofluorescence staining to detect the distribution of CD19 and IL-10 in thymus tissues. Thymoma patients without MG mainly display the types A and AB of thymoma, whereas the thymoma patients with MG mainly display type B (B1, B2 and B3) thymoma; AChR-Ab in Tm + MG group was the highest, with the progress of the disease, the percentage of Breg/CD19^+^B cells increased and B10/CD19^+^B cells decreased (*p* < 0.05); ROC curve showed that B10 had the greatest significance for the clinical directivity of Tm+MG and cut-off point = 0.55%; in accordance with the Con, Tm and Tm+MG group, the content of CD19^+^IL-10^+^B10 cells increased gradually (*p* < 0.05); meanwhile, the gene and protein expression levels of CD19 and IL-10 gradually increased in the same way. It is concluded that with the progress of thymoma, the infiltration of Breg in tumour tissue increases; however, as the severity of MG increases, the function of Breg (B10 cell) in peripheral blood decreases and the cut-off point is 0.55%.

## INTRODUCTION

Thymoma is a tumour originating from thymic epithelial cells and often associated with various autoimmune diseases mediated by T cells, and myasthenia gravis (MG) is one of the most common complications of them, which incidence can be as high as 40% [1]. Currently generally considered that the most common Breg cell phenotype in human peripheral blood is CD19^+^CD24^+^CD38^+^, and the functional Interleukin-10 (IL-10)-secreting Breg cells are called B10 cells. In recent years, with the researches of Breg, even B10 cells and tumor-related immune microenvironment gradually carried out, there is growing evidence that, B10 cells play a key role in the pathogenesis and regulation of thymoma with related autoimmune diseases, especially in MG [2]. Thus, we regarded the CD19^+^CD24^+^CD38^+^B cells in peripheral blood as “Breg cells”, the CD19^+^CD24^+^CD38^+^ IL-10^+^B cells in the peripheral blood and the CD19^+^IL-10^+^B cells in the thymus tissues as “B10 cells” in our experiment. This study investigated the characteristics of B10 cell in disease diagnosis, assessment of the severity and prognosis of diseases in patients with thymoma complicated by MG, and explored a new approach for the theory and practice in this field.

## RESULTS

### General condition and classification of clinical patients

All the patients enrolled were classified according to the pathological types of tissue specimens. From Table 1 and Figure 1, we could find that the thymoma patients without MG mainly display the types A and AB of thymoma, whereas the thymoma patients with MG mainly display type B (B1, B2 and B3) thymoma.

**Table 1:** General situation of patients enrolled

	Con (*n*)	Tm (*n*)	Tm+MG (*n*)	Total (*n*)
Thymic cyst (*n*)	5	0	0	5
Thymoma type A (*n*)	0	17	5	22
Thymoma type AB (*n*)	0	40	12	52
Thymoma type B1 (*n*)	0	12	31	43
Thymoma type B2 (*n*)	0	4	16	20
Thymoma type B3 (*n*)	0	3	11	14
Total (*n*)	5	76	75	156

**Figure 1:** General situation of patients enrolled All the patients enrolled were classified according to the pathological types of tissue specimens. From Figure 1we could see that the thymoma patients without MG mainly display the types A and AB of thymoma (17/22 patients without MG for types A thymoma; 40/52 patients without MG for types AB thymoma), whereas the thymoma patients complicated with MG mainly display type B (B1, B2 and B3) thymoma (31/43 patients with MG for type B1 thymoma; 16/20 patients complicated with MG for type B2 thymoma; 11/14 patients complicated with MG for type B3 thymoma).

### Comparison of preoperative immunological parameters

We compared the immunological parameters, including IgG, IgM, acetylcholine receptor antibody (AChR-Ab), B10/CD19^+^B cell, Breg/CD19^+^B cell, CD19^+^B cell/PBMC, of all enrolled pre-operative patients of the different groups. In this article, we regarded “CD19^+^CD24^+^CD38^+^ B cell” as Breg, and “CD19^+^CD24^+^CD38^+^IL-10^+^ B cell” as B10 cell.

The result shows that IgG and IgM had of the three groups did not significant differs (Table 2); AChR-AB significantly differed between the Tm and Tm+MG groups (Table 2, Figure 3A). Moreover, although CD19^+^B/PBMC levels did not significantly differ in the three groups (Table 2, Figure 3B), Breg/CD19^+^B cell (%) and B10/CD19^+^B cell (%) of Tm+MG group significantly differed to that of the two other groups (Table 2, Figure 2). In Tm+MG group, the percentage of Breg/CD19^+^B cell increased (Figure 3C), while the percentage of B10/CD19^+^B cell decreased (Figure 3D) (*p* < 0.05), indicating that with the emergence or exacerbation of MG symptoms, B cell count in the peripheral blood did not significantly change, but AChR-Ab content and the percentage of Breg cells increased while the percentage of B10 cells decreased.

**Table 2:** Comparison of immunological parameters before operation

	IgG (g/L)	IgM (g/L)	AChR-Ab (ng/ml)	**B10/CD19**^+^**B cell (%)**	**Breg/CD19**^+^**B cell (%)**	**CD19**^+^**B cell/ PBMC**
Con group	14.90 ± 0.860	1.05 ± 0.516	0.60 ± 0.092	1.32 ± 0.179	2.33 ± 1.05	7.13 ± 0.48
Tm group	15.16 ±1.545	1.31 ±0.392	0.59 ± 0.060	1.22 ± 0.332	2.54 ± 0.12	7.03 ± 0.55
Tm+MG group	14.83 ± 1.365	1.29 ± 0.329	0.79 ± 0.078*	0.53 ± 0.145*	3.15 ± 0.58*	7.87 ± 0.23

*indicated *p* < 0.05 and have statistically significant difference.

**Figure 2:** Flow cytometry analysis of peripheral blood Breg cells Peripheral blood cells were stained with the indicated fluorescent-antibodies against. The frequency of each type of cells was determined by flow cytometry. In addition, peripheral blood cells were stained with PE-Cy7-conjugated anti-human CD19, APC-conjugated anti-human-CD24, FITC-conjugated anti-human-CD38, then, fixed and permeabilized, followed by intracellular staining with PE-conjugated anti-human-IL-10. The numbers of each type of cells were calculated in different groups.

**Figure 3:** Comparison of related immune parameters (**A**). Concentration of AChR-Ab in different groups; (**B**). The percentage of CD19^+^B cell/PBMC in different groups; (**C**). The percentage of Breg/CD19^+^B cell in different groups; (**D**). The percentage of B10/CD19^+^B cell in different groups.

### Immunological markers for clinical recognition of thymoma with MG

We used generalized clinical remission (CSR+PR+MM+I) as the end of the study. Among the four indicators, B10 and AChR-Ab showed the largest AUC, and Breg > AChR-Ab, indicating that B10 percentage had the greatest significance for the clinical significance for the thymoma with MG (Figure 4, Table 3).

**Figure 4:** ROC curve of B10 percentage, AChR-Ab, IgM, IgG In Figure 4, we could see the B10 percentage and AChR-Ab showed the largest AUC (0.748 and 0.658 respectively), and the former had statistical significance (*p* = 0.003). From Figure 4, we could indicated that the B10 percentage had the greatest significance for the clinical significance for the thymoma with MG.

**Table 3:** Immunological markers for the clinical recognition of thymoma with MG

		IgG	IgM	AChR-Ab	**B10 / CD19**^+^**B cell**
Area		0.498	0.591	0.658	0.748
*p* value		0.985	0.280	0.059	0.003*
Progressive 95% confidence interval	upper	0.681	0.718	0.812	0.860
	Lower	0.316	0.463	0.504	0.636

*indicated *p* < 0.05 and have statistically significant difference.

### Calculation of B10 cut-off point and relationship between B10 and MG classification based on MGFA

On the basis of the sensitivity and specificity values of ROC curve, we obtained a cut-off point for B10/CD19^+^B cell of 0.55% (0.692 for sensitivity and 0.748 for specificity). By combining this cut-off point with that of B10, we used the MGFA classification of MG to evaluate the significance of B10 in MG.

We found that in 75 patients with MG, percentage of B10 > 0.55% was mainly about the patients of type II and type III, percentage of B10 < 0.55% was mainly about the patients of type IV and type V (Table 4, Figure 5).

**Table 4:** The MGFA classification of MG combined with cut-off point of B10

	Type I (*n*) (%)	Type II (*n*) (%)	Type III (*n*) (%)	Type IV (*n*) (%)	Type V (*n*) (%)	Total
**>** cut-off point	0 (0.00)	11 (14.67)	19 (25.33)	4 (5.33)	0 (0.00)	34
≤ cut-off point	0 (0.00)	0 (0.00)	3 (4.00)	29 (38.67)	6 (8.00)	41
Total	0	11	22	33	6	75

**Figure 5:** The MGFA classification of MG combined with cut-off point of B10 By combining this cut off point with that of B10, we used the MGFA classification of MG to evaluate the significance of B10 in MG.

### Comparison of the distribution of B10 in different groups of thymus mass tissues

Based on the results of pathological analysis, the patients were divided into Con, Tm and Tm+MG groups. The thymus specimens of all patients were subjected to double immunofluorescence staining, and then we performed semi-quantitative analysis by Software Tissuequest 4.0.1.0140.

The results of the semi quantitative analysis show that, with the development of thymoma (Tm group) and the appearance of MG (Tm+MG), the infiltration of CD19^+^IL-10^+^ B10 cells increased gradually (Figure 6). Through the Software Tissuequest 4.0.1.0140, we could also found that the fluorescent spot area of CD19 and IL-10 was getting bigger (Figure 7).

**Figure 6:** Double fluorescence staining of CD19 and IL-10 in thymus tissues Legend: blue - nucleus; green - CD19 (located in cell membrane), red - IL-10 (located in nucleus or cytoplasm).

**Figure 7:** The semi quantitative analysis of the percentage of CD19^+^IL-10^+^B10 cells according to the double fluorescence staining by Software Tissuequest 4.0.1.0140

We also made the semi quantitative analysis of the distribution of B10 cells in thymus (Supplementary Figure 1) from which we could see that the spots number of CD19 (Supplementary Figure 1A) and IL-10 (Supplementary Figure 1B) were the most in Tm+MG group and least in Con group. Thus, it was represented an increase in the infiltration of CD19^+^IL-10^+^ B10 cells in tumour tissues.

### Comparison of the gene and protein expression levels of CD19 and IL-10 gene in CD19^+^B cells

To evaluate and detect the functional antibody of IL-10 secreted by CD19^+^B cells, we used the MACS technology in separating CD19^+^B cells from thymus tissues. Real-time PCR and Western blot assay were used to detect the gene and protein levels of CD19 and IL-10.

The protein (Figure 8A–8C) and gene (Figure 8D, 8E) expression levels of CD19 and IL-10 gradually increased in the Con group, Tm group and Tm + MG group, and significant differences were observed compared to the Con group (*p* < 0.05).

**Figure 8:** The quantitative analysis of protein and gene expressions of CD19 and IL-10 (**A**, **B** and **C**) showed the protein expression levels of CD19 and IL-10 in different groups; (**D** and **E**) showed the gene expression levels of CD19 and IL-10 in different groups. (A) showed the protein expression of CD19 and IL-10 by western-blot; (B) and(C) showed the protein of CD19 and IL-10 was the highest in the Tm+MG group, and the lowest in the Con group. The relative expression of gene levels of CD19 and IL-10 in (D) and (E) had the same trend as those in (B) and(C), indicating that gene of CD19 and IL-10 was the highest in Tm + MG group and the lowest in Con group.

## DISCUSSION

Thymoma is a tumour originating from thymic epithelial cells; it is potentially malignant and one of the most common human tumours associated with autoimmune diseases; moreover, thymoma is closely related to MG [3]. Conversely, 75% MG patients show abnormal thymus gland and 15% of these cases are thymoma [4]. In clinics, we found that thymoma with MG is more complex compared with simple MG, and sometimes it promotes the incidence of MG in patients after thymectomy. Currently, relevant clinical examination indicators, such as AChR-Ab, IgM and IgG, and even the complement tests C3 and C4 cannot directly and specifically reflect the severity of MG. Thymoma with MG is caused by a disorder in the autoimmune system, and this disease is complex; a new indicator must be identified to assess its progression, severity and prognosis. Analysis of thymoma patients with MG showing complicated condition and long-term poor prognosis revealed the following: (1) patients with thymoma showed a high AchR-Ab antibody titer, which decreased slowly post-operation. (2) thymoma patients with MG often display secretion of various autoantibodies, such as RyR-Ab. (3) incidence of thymoma may course the immune system more complex. Studies have reported that the symptoms are possibly more serious post operation in some patients with thymoma resection; new MG symptoms may even emerge, likely resulting in secretion of some cytokines that inhibit autoimmune inflammatory reaction and possibly inducing the onset of MG symptoms after thymoma resection [5].

In recent years, an increasing number of researchers has found that a new subtype of B cells that secretes IL-10 and transforms growth factor beta (TGF- beta) and other immunosuppressive factors, and then inhibits the immune response; these cells are known as regulatory B cell (Breg), which has the function of IL-10 secretion is known as B10 cells [6–7]. Breg and B10 occupy important roles in various diseases, involved in occurrence of disease, progression and prognosis and involved in other physiological processes [8]. Compared with the regulatory T cell (Treg), which displays a specific phenotype (CD4^+^CD25^+^Foxp3^+^), Breg cells exhibit a diverse phenotype, and no specific phenotype has been found. Basic research has currently recognized the following Breg phenotypes: CD19^+^CD24^+^CD38^+^, CD19^+^CD5^+^CD1d^+^, CD19^+^CD24^+^CD27^+^, CD19^+^CD38^+^CD1d^+^IgM^+^CD147^+^, CD25hiCD71hiCD73lo and CD27intCD38hi [9]. Given the recent introduction of the concept of “tumour immunity,” studies have found that tumour progression is associated with the infiltration of B cells. Breg inhibits progression of autoimmune diseases and inflammatory diseases by secreting IL-10 or TGF- beta [10–11]. Studies on tumour immunity have found the immune regulatory effect of Breg on T cells and NK cells in immune-related tumour microenvironment [12], similar to the findings on Breg in related studies on autoimmune diseases, inflammatory responses and infections. Thus, Breg builds a bridge between immune regulation and tumours [13–14]. Research has shown that with growth of solid tumours, invasion or metastasis, an increasing number of Breg cells infiltrate tumour tissues [15], indicating that Breg is involved in tumour related immune microenvironment [16–17].

In order to investigate the role of B10 to thymoma complicated with myasthenia gravis, we retrospectively analysed 156 patients with thymoma, and they were divided into Con group, Tm group, and Tm+MG group.

Based on the clinical indicators in the peripheral blood samples of the patients in the three groups, CD19^+^B cell/PBMC, Breg/CD19^+^B cell, B10/CD19^+^B cell, AChR-Ab, IgG and IgM levels did not significantly differ between the Con and Tm groups. Compared with Tm and Con groups, Tm+MG group displayed a significantly higher AChR-Ab and percentage of Breg/CD19^+^B cell and lower percentage of B10/CD19^+^B cell. In thymoma with MG, autoimmune inflammation was activated accompanied by emergence of MG or the MG symptoms increased, B cell count in peripheral blood did not significantly change and AChR-Ab content and Breg percentage increased with a decrease in the percentage of B10; this result indicated that the function of B10 decreased or consumption increased.

We used the MGFA intervention status to classify the patients, and the recovery of MG patients was followed up for 2 years; the generalized clinical remission (CSR+PR+MM+I) served as the study end point of efficacy assessment. We subsequently obtained the ROC curve of the four clinical parameters and then calculated the area under the curves. The areas of B10/CD19^+^B cell and AChR-Ab were the two highest indexes, and the area of B10/CD19^+^B cell is larger than AChR-Ab, illustrating that B10 demonstrated higher clinical accuracy in recognizing thymoma with MG. Moreover, we obtained the most sensitivity and specificity point to be the best value of 0.55% and as the cut-off point of B10/CD19^+^B cell.

All patients underwent thymectomy, and the specimens were preserved for semi quantitative (immunofluorescence double staining) and quantitative protein detection (Western blot) of CD19 and IL-10. The thymus tissue of Tm+MG group displayed extensive infiltration of CD19^+^IL-10^+^ B10 cell, and the infiltration degree was significantly higher in this group than in Con and Tm groups. As showed in Table 1, 57 patients (57/76, 75%) displayed benign thymoma (types A and AB) and 19 patients (19/75, 25%) had malignant thymoma (types B1, B2 and B3) in Tm group; whereas in Tm+MG group, 17 cases (17/75, 22.67%) showed benign thymoma (types A and AB) and 58 patients (58/75, 77.33%) displayed malignant thymoma (types B1, B2 and B3), demonstrating that the higher the degree of progress of thymoma, the greater the likelihood of development of thymoma with MG. As revealed by protein quantitative analysis, with the progress of pathological types of thymoma, infiltration of B10 in the thymus increased significantly, corresponding with greater tendency of MG complication. Finally, in view of the level of IL-10 secreted by B10 in thymus tissues, CD19^+^B cells were purified by MACS, and after detection through real-time PCR and Western blot assay, the expression levels of CD19 and IL-10 in Tm+MG group were significantly higher than those in the Con and Tm groups, demonstrating that B10 was involved in thymoma progression and possibly involved in pathogenesis of thymoma with MG.

Based on semi quantitative comparison of B10/CD19^+^B cell in peripheral blood and thymus tissue, we seemingly came to the contradictory conclusions. In fact, it is not unreasonable. We observed that the percentage of Breg/CD19^+^B cell in peripheral blood and B10/CD19^+^B cell in thymus tissue significantly increased in the Tm+MG group compared with that in Con and Tm groups, but the percentage of B10/CD19^+^B cells in the peripheral blood decreased compared with that in the two other groups. We considered the following two reasons:

On one hand, recent literature suggests that the same cell or cytokine may play a distinct role in different microenvironments [18]. Clinical animal experiments on tumour immune microenvironment have shown that through infiltration in tumour tissues, Breg secreted IL-10 or TGF-beta to suppress the body’s immune response to tumour cells and promoted tumour cells’ immune escape [19–20]. Shi [21] have found secretion of IL-10 and TGF-beta by Breg increased significantly in patients with esophageal cancer compared with that in control group, and TGF-beta significantly decreased after operations and the number of CD19^+^IL-10^+^B cell increased compared with that in pre-operation. In our experiment, infiltration of Breg in thymoma tissues showed similar results. With thymoma progression, B10 infiltration in tumour tissue increased along with the increase in incidence tendency of MG, indicating that B10 promotes the development of thymoma complicated with MG.

On the other hand, IL-10 enhances DNA synthesis and amplification in B cells, induces differentiation of B cells into plasma cells and secretes IgM and IgG. Studies have suggested that the effect of IL-10 is mediated by DCs or macrophages by promoting the expression levels of CXCL-13 and SLAM (signalling lymphocytic activation molecule) to recruit and activate peripheral blood B cells [22]. In our experiment, increase in percentage of Breg/CD19^+^B cell was also observed. While with the emergence of MG and aggravation of the symptoms, the function of secretary of IL-10 from Breg decreased or the percentage of B10/CD19^+^B cell decreased, suggesting the decrease in Breg’s function or the increase in B10’s consumption, consistent with the result of Sun F [23].

Our result showed that that with the emergence of MG, the percentage of B10/CD19^+^B cell decreased, whereas the percentage of Breg/CD19^+^B cells and the amount of AChR-Ab increased. Thus, we can infer that ① the degree of infiltration of B10 cells in thymus tissue was gradually increased in Con group, Tm group and Tm+MG group, and thymoma may increase the growth of tumour by increasing the infiltration of B10 cells in tumour microenvironment, and its enrichment is positively correlated with the progression of thymoma and the tendency of thymoma complicated with myasthenia gravis; ② Combination of the ratio of B10/CD19^+^B cells in the peripheral blood of Tm+MG group was lower than that in the other two groups, while the percentage of Breg/CD19^+^B cells and the AChR-Ab content increased, we can infer that B10 cells are likely to stimulate peripheral blood B cells to secrete AChR-Ab, and which can stimulate the differentiation of B cells to Breg at the same time. However, during the process of MG, the cells function decreased or consumed, which may lead to decrease of the proportion of B10/CD19^+^B cells. Of course, the pathogenesis of thymoma complicated by autoimmune diseases is very complex, and it is not caused by a single factor. Thus, further research is needed to clarify the specific mechanism of the regulatory effect of Breg on thymoma with MG.

Our experiments came to a conclusion of B10 in tumour associated immune microenvironment and are closely related to the pathogenesis and progression of thymoma with MG, that is to say, B10 promotes the progress of thymoma and activates the pathogenesis of thymoma with MG; with the progress of thymoma, B10 cells infiltration in tumour tissue increases while as the severity of MG increases, the function of Breg in peripheral blood is inhibited. Combined with the cut-off value, we have made an important supplement to the theoretical basis for clinical application of Breg.

## MATERIALS AND METHODS

### Clinical data collection

This study was approved by the Ethics Committee of Tianjin Medical University Cancer Institute and Hospital. All of the patients signed the consent forms. This experiment enrolled patients diagnosed with thymus mass in the Lung Cancer Department of Tianjin Medical University Cancer Institute and Hospital within from April 2010 to March 2015. Inclusion Criteria: (a) patients diagnosed with thymoma according to the NCCN (2016); (b) age range of patients is 18–60 years; (c) complicated with or without myasthenia gravis (MG); and (d) all the patients enrolled in the study were treated with thymus mass resection under thoracoscopic or through median sternotomy incision by general anesthesia. Exclusion Criteria: (a) hypertension, diabetes, coronary heart disease and other chronic diseases and (b) complicated with other autoimmune diseases, such as systemic lupus erythematosus, scleroderma, pemphigus and pemphigoid. This study enrolled five cases of thymic cyst as control.

This experiment enrolled 156 patients, 72 of which were males (average age: 39.2 ± 7.59 years) and 84 were females (average age: 42.8 ± 6.87 years). Among these cases, 5 were thymic cyst (Con), 76 were thymoma (Tm) and 75 were thymoma complicated with MG (Tm+MG). The pathological types were as follows: 5 were thymic cyst; 27 were Type A thymoma, 52 were Type AB thymoma, 43 were Type B1 thymoma, 20 were Type B2 thymoma and 14 were Type B3 thymoma.

The patients complicated with MG were treated with regular oral pyridostigmine (120 mg Tid to Qid), and then the prednisone tablets would be given under the poor control of the symptom of MG. All of the patients underwent thymectomy, and the timing of operation was the symptoms improving significantly and the dose of prednisone was lower than 20mg per day for the patients with MG.

A standardized follow-up file was established, and drug dosage was gradually reduced based on the improvement in symptoms. The use of drug was gradually stopped when the symptoms of MG disappeared for more than 6 months; however, the patients would need to receive drug re-treatment if the symptom relapses.

### Evaluation standard

#### Diagnostic evaluation criteria

Clinical severity of MG patients was assessed according to the clinical classification criteria of Myasthenia Gravis Foundation of America (MGFA) [24]. The follow up period was 2 years, and MGFA score was used as index to evaluate the effectiveness of the operation. The evaluation was divided into five classes: Class I: Weakness of any ocular muscle, and possible weakness of eye closure. All other muscles show normal strength. Class II: Mild weakness affecting muscles other than the ocular muscles; ocular muscle weakness of any severity is possibly experienced. Class III: Moderate weakness affecting muscles other than ocular muscles; ocular muscle weakness of any severity is possibly experienced. Class IV: Severe weakness affecting muscles other than ocular muscles; ocular muscle weakness of any severity is possibly experienced. Class V: Defined as intubation with or without mechanical ventilation, except when employed during routine postoperative management.

### Criteria for prognostic evaluation

Prognostic assessment using the MGFA post-intervention status, including complete stable remission (CSR), pharmacological remission (PR), minimal manifestations (MM), improved (I), unchanged (U), worse (W), exacerbated (E) and death of MG (D). In this study, generalized clinical remission (CSR+PR+MM+I) was used as an indication of the end of the study.

### Specimen processing and experiment methods

### Specimen processing

For blood samples, venous blood (4 ml) extracted from all of the patients before breakfast prior to the operation, and detected the related immune parameters. For tissue specimens, specimens obtained during operations were routinely examined by pathologists. Fresh thymus tissue was digested with Collagenase IV, and the rest of the specimens were placed in formalin or stored in a refrigerator at ‒80°C.

### Flow-cytometry

Venous blood samples (4 ml) were extracted for peripheral blood mononuclear cells (PBMC) through density gradient centrifugation with Ficoll separation solution, subsequently stimulated with PMA + ionomycin for 4–6 h. Re-suspended in 300 ul phosphate-buffered saline (PBS) and stained with PE-Cy7-conjugated anti-human CD19, APC-conjugated anti-human-CD24, FITC-conjugated anti-human-CD38, then, fixed and permeabilized, followed by intracellular staining with PE-conjugated anti-human-IL-10 (eBioscience Company, USA). Flow-cytometry data were acquired using a flow cytometry on a BD FACSCalibur™ (BD Biosciences, San Jose, USA). At least 20,000 events were collected for each analysis. All data were further analyzed by FlowJo software (Tree Star).

### Enzyme linked immunosorbent assay (ELISA)

Fasting venous blood samples were collected from individual patients before surgery. The concentrations of serum IgG (g/L), IgM (g/L), AChR-Ab (ng/ml) in individual patients were tested by enzyme-linked immunosorbent assay (ELISA) (Human IgG, IgM and AChR-Ab ELISA Kit , bought from Abcam Company, Britain) .

### Double immunofluorescence staining

The tissues slices were incubated with a polyclonal rabbit anti-IL-10 (bought from Abcam Company, Britain) and mouse monoclonal anti-CD19 (bought from Abcam Company, Britain) antibodies for 16 hours under 4°C at a dilution of 1:300 and 1:100, respectively. Subsequently, the slides were incubated with a mixture of secondary antibody for IF. Both secondary antibodies were used at a dilution of 1:100. Then, CD19/IL-10 Double immunofluorescence staining was observed under Confocal fluorescence microscopy (Olympus, Center Valley, PA, USA), and we performed semi-quantitative analysis by Software Tissuequest 4.0.1.0140. We stained the nucleus with DAPI, spot number of CD19 and IL-10 was collected by the software and DAPI spots number was seemed as reference. We calculated the spots number of CD19 and IL-10/spots number of DAPI, so as to obtain the relative cell counts of CD19 and IL-10 in thymus tissue of different groups.

### MACS MicroBeads

Fresh thymus tissue was digested with Collagenase IV, and single cell suspension was prepared by using 200 mesh sieves. Human B cells were labeled with microbead-conjugated CD19 mAb according to the manufacturer’s instructions (CD19 MACS MicroBeads, bought from Miltenyi Biotec Company, Germany) and incubated for 30 min (all solutions were ice-cold and all incubations were performed at 4°C and protected from light). CD19^+^ Microbead-labeled T cells were washed, resuspended in PBS-0.5% BSA, passed over a MACS preseparation filter, and separated in MACS separation columns that were exposed to a magnetic field. Sorted CD19^+^B cells were washed and subsequently flushed from the column with PBS–0.5% BSA. Last, sorted T cells were counted and prepared for Real-time PCR and Western-blot assay.

### Real-time PCR

Total RNA was isolated from CD19^+^B cells purified by MACS MicroBeads, using TRIzol Reagent (Goldenbridge Biotech, Beijing, China), according to the manufacturer’s instructions. After digestion with DNase 1, the RNA samples were reverse transcribed into cDNA using oligo(dT) primers (Takara, Beijing, China) and TransScrinpt RT/RI/Enzyme Mix (Takara). The relative levels of CD19, IL-10 mRNA transcripts to the control glyceraldehyde 3-phosphate dehydrogenase (GAPDH) were determined by quantitative RT-PCR using SYBR green PCR master mix buffer (Takara) and specific primers. The primers were designed and synthesized by Sangon Biotech Company (Shanghai, China). The sequences of primers were sense 5′-TCTTCCTCACCCCCATGGAA-3′ and antisense 5′- ACTGCAGCACAGCGTTATCT-3′ for CD19; sense 5′- TTCCAGTGTCTCGGAGGGAT-3′ and antisense 5′- GCTGGCCACAGCTTTCAAGA-3′ for IL-10; sense 5′-GAAGGTGAAGGTCGGAGTC-3′ and antisense 5′-GGGTGGAATCATATTGGAAC-3′ for GAPDH. The PCR amplification was carried out at 94°C for 3 min and subjected to 35 cycles of 94°C for 30 sec, 56–58°C for 30 sec, and 72°C for 1 min, followed by a final extension at 72°C for 5 min. The relative levels of target gene expression were normalized to the GAPDH and analyzed by 2^-∆∆Ct^.

### Western-blot assay

Protein extracts of CD19^+^B cells purified by MACS MicroBeads were electrophoresed on 10% SDS polyacrylamide gels and transferred to nitrocellulose membranes. Membranes were blocked with 5% non-fat dried milk and incubated for overnight with an appropriate primary antibody: CD19 and IL-10 (bought from Abcam Company, Britain), followed by the horseradish peroxidase-conjugated secondary antibody. The immunocomplexes were visualized using the chemiluminescence phototope-horseradishperoxidase kit. GAPDH was used to ensure equivalent protein loading. The integrated density of the band was quantifed by ImageJ sofware.

### Statistical analysis

Data were analysed using the SPSS 19.0 statistical software. Independent sample *t*-test was used for continuous variables, and data were analysed by chi-square test or exact probability method, data are representative charts and expressed as the mean ± SD of each group of patients. The Kaplan–Meier method was used for single factor analysis of generalized postoperative clinical remission. ROC curve was used to evaluate the clinical significance of each index. *P* < 0.05 indicated statistical significance.

## SUPPLEMENTARY MATERIALS FIGURE



## Abbreviations

(MG): Myasthenia gravis
(MGFA): Myasthenia Gravis Foundation of America
(Breg): regulatory B cell
(IL-10): Interleukin-10
(AChR-Ab): acetylcholine receptor antibody
(ELISA): enzyme linked immunosorbent assay
(PBMC): peripheral blood mononuclear cells
(CSR): complete stable remission
(PR): pharmacological remission
(MM): minimal manifestations
(I): improved
